# Effect of Functional Electrical Stimulation on Gait Parameters in Children with Cerebral Palsy: A Meta-Analysis

**DOI:** 10.1155/2022/3972958

**Published:** 2022-09-22

**Authors:** Qiantao Zhu, Guanchen Gao, Kaijiang Wang, Jingjing Lin

**Affiliations:** ^1^Department of Rehabilitation Medicine, Hainan Western Central Hospital, Danzhou 571700, China; ^2^Department of Neurosurgery, Danzhou People's Hospital, Danzhou 571700, China; ^3^Department of Rehabilitation, Sanya Traditional Chinese Medicine Hospital, Sanya 572000, China

## Abstract

**Objective:**

At present, there are controversies on the effectiveness of functional electrical stimulation devices in gait improvement in the clinic, and the results reported in limited literature are contradictory. This paper summarizes and analyzes the relationship between functional electrical stimulation treatment and gait parameter changes in children with cerebral palsy, thus exploring the above controversies' results.

**Methods:**

Two researchers conducted a detailed search of the literature from the establishment of the database to June 2022. Literature retrieved from databases, including PubMed, Embase, Ovid, Cochrane Library, and Web of Science and the search process followed the principles of Cochrane. The search keywords were “cerebral palsy”, “functional electrical stimulation”, “gait”, or “walk”. Gait and balance parameters were extracted from the literature. Gait parameters, such as walking speed and step length, were included in the meta-analysis. The study used standard mean difference (STD) and 95% confidence interval (CI) to calculate the mean difference between the two groups. The statistic *I*^2^ was used to evaluate the heterogeneity between the evaluation studies. Begg's test detected publication bias and the funnel chart was used for visual analysis. Furthermore, Review Manager software was used to make a risk bias map for literature publication bias analysis.

**Results:**

9 literatures were included in the analysis, with a total of 282 children with cerebral palsy, including 142 patients in the functional electrical stimulation treatment group and 140 patients in the comfort treatment, general nursing, or other physical therapy. The randomization scheme and result report used in most studies were low risk, which was important for the credibility of this study. Most studies have limitations in the blinding method of participants and subjects, and most of them were single-blind studies, which might have a high risk. The results showed that functional electrical stimulation could increase the walking speed of children with cerebral palsy (SMD = 0.82, *P* < 0.0001) and increase the walking step length of children with cerebral palsy (SMD = 1.34, 95%CI = 1.07, 1.60, *Z* = 9.91, *P* < 0.0001). Funnel plot analysis showed that the literature distribution was uniform and symmetrical, and Begg's test showed no publication bias in included literature.

**Conclusion:**

This study compared the effects of the functional nerve stimulation treatment group and control group on improving gait parameters of children with cerebral palsy. The results indicated that functional nerve stimulation treatment could increase the gait speed and step length of children with cerebral palsy, which could improve the walking of children with cerebral palsy. Furthermore, this study needs more research data to support our findings. The results of this study might better guide the clinical practice and better use of health as well as financial resources.

## 1. Introduction

Cerebral palsy (CP) is a common neurological disease caused by nonprogressive disorders in the development of the central nervous system. The clinical symptoms include a series of motor and posture disorders [1]. Children with cerebral palsy usually show obstacles in neuromotor, musculoskeletal, and sensory systems, resulting in muscle strength loss and dysfunction. Furthermore, cerebral palsy can impair motor control and hinder various motor skills required by children's daily activities, such as walking [2, 3].

As patients grow up, the gradual increase in weight, muscle strength, and involuntary muscle contraction cause abnormal biomechanics, thus leading to abnormal walking and gait patterns in children [4]. However, walking and gait are the abilities necessary for moving and exploring the environment. These problems bring the most severe functional impairment and the highest frequency of abnormalities in children with cerebral palsy, which greatly challenges clinical rehabilitation and intervention [5, 6]. Therefore, defining gait parameters is particularly important because they reflect the changes in the physical structure and function of children with cerebral palsy [7]. The improvement of gait parameters enhances motor function, allowing children with cerebral palsy to explore different ground environments and improve social interaction and participation, which has a positive impact on clinical rehabilitation and intervention [8].

Functional electrical stimulation (FES) is a kind of neural stimulation device which has been widely used in clinical rehabilitation and intervention. Currently, it is mainly used to stimulate muscles or nerves with impaired motor control ability to enhance the control and execution of functional actions [9]. FES is applied in the gait cycle mainly by stimulating appropriate muscle groups, such as the common peroneal nerve, to facilitate the ankle joint dorsiflexion and prevent the foot from falling. Therefore, FES can correct the gait swing state deviation and improve the walking ability [10]. In clinical rehabilitation, FES is mainly used to increase muscle strength, reduce muscle spasms, and improve exercise mode. Moreover, the FES device is small in size and easy to use, thus it is widely used in the clinic [10].

Currently, limited data support the role of FES in supporting walking by improving muscle strength and reducing muscle spasms [11]. Meanwhile, current literature data are based on clinical experiences or case reports, which lack evidence-based data on the walking gait improvement of FES. At the same time, there are controversies on the effectiveness of functional electrical stimulation devices in gait improvement in the clinic, and the results of limited literature reports are contradictory. For example, Armstrong et al. reported in a randomized controlled trial of 21 participants that the gross motor function measurement (GMFM) of the intervention group undergoing FES cycle training was superior to that of the routine nursing control group [12]. In contrast, Ozen et al. conducted a randomized controlled trial of 25 participants. They observed significant improvements in the evaluation of exercise ability in the FES cycle training group and the sham stimulation group, including GMFM measurement. However, the two groups had no statistical differences [13]. Due to the contradiction and inconsistency of clinical evidence, a high-quality systematic review and meta-analysis are required.

In this study, we summarized and analyzed the relationship between functional electrical stimulation and gait parameter changes in children with cerebral palsy to explore the controversial results. More updated clinical experimental studies were included in our research to ensure that the analysis results had all current experimental evidence, thus obtaining more accurate results and avoiding bias.

## 2. Materials and Methods

### 2.1. Literature Search Strategy and Inclusion and Exclusion Criteria

The two researchers conducted a detailed search of the literature from the beginning of the database to June 2022. The search process followed the principles of Cochrane, and the following databases were searched: PubMed, Embase, Ovid, Cochrane Library, and Web of Science. The search keywords were “cerebral palsy”, “functional electrical stimulation”, “gait”, or “walk”. The other 2 researchers collected literature that met the criteria after reading the titles and abstracts. Disparities arising from literature retrieval were resolved through negotiation and discussion.

The inclusion criteria were as follows: (1). The randomized controlled trial included the FES application test group and corresponding control group, and the control group could not be another electrical stimulation group; (2): The subjects were children with cerebral palsy under 18 years old; (3): During walking, the muscles were treated with functional electrical stimulation; (4): Detailed quantitative gait analysis data were provided; (5): Only English articles were analyzed.

Exclusion criteria were as follows: (1): Nonrandomized controlled trials, including prospective trials or retrospective studies, or it was impossible to determine whether the literature was a randomized controlled trial; (2): Other percutaneous electrical stimulation studies; (3): Gait disorder caused by other neurological diseases; (4): Adult patients.

### 2.2. Document Data Extraction and Analysis

Gait and balance parameters were extracted from the included literature. Gait parameters, such as walking speed and step length, were included in the meta-analysis. Other parameters were not included in the meta-analysis as the data identified in the literature.

Meta-analysis was performed using Review Manager software (version 5.4 of the Nordic Cochrane Centre, Copenhagen, Denmark). Forest maps were established to assess the data differences between the FES test group and the control group. The study used stand error of mean (STD) and 95% confidence interval (CI) to calculate the mean difference between the two groups. The statistic *I*^2^ was used to assess the heterogeneity between the evaluation studies. The random effect model was used when *I*^2^ was greater than 50% and the heterogeneity was significant. Otherwise, the fixed effect model was used. Publication bias was detected by Begg's test and the funnel chart was conducted for visual analysis.

### 2.3. Document Quality Evaluation

By following the analysis guidelines provided by the Cochrane Library, the bias risk analysis tool of Review Manager software was used to prepare the risk bias map. The bias risk analysis included the generation of random sequence, the concealment of the allocation scheme, the blinding of participants and subjects, the blinding of results evaluation, the integrity of results, the bias of results report, and other biases. The bias risk included three levels, namely, low, high, and unclear. The results were marked with red, green, and yellow color blocks.

## 3. Results

### 3.1. Retrieval Results and Literature Quality Evaluation

The document search and screening process is shown in Figure 1. In this study, a total of 897 articles about the effect of functional electrical stimulation on gait parameters of children with cerebral palsy were retrieved from the database. After screening according to the above literature inclusion and exclusion criteria, 9 literatures [12–20] were finally included in the analysis, with a total of 282 children with cerebral palsy. Among them, 142 patients were divided into the functional electrical stimulation treatment test group, and 140 patients were included in the control group, treating with comfort treatment, general nursing, or other physical therapy. To reduce the heterogeneity of the study, FES combined with other treatments such as botulinum toxin treatment was excluded. In this paper, the functional electrical stimulation treatment group was taken as the experimental group, and the comfort treatment, general nursing, or other physical therapy groups were taken as the control group. The 9 included studies were all subject to literature quality assessment. Figures 2 and 3 are the summaries of bias risk and the detailed analysis bar chart of bias risk of each included document. Each study had its own high risk and indeterminate situation. In general, the randomization scheme and results report used in most studies are low-risk, which was critical to this study's credibility. Most studies have limitations in the blinding method of participants and subjects, and most of them were single-blind studies, which might have a high risk.

### 3.2. Effect of Functional Electrical Stimulation on Walking Speed of Children with Cerebral Palsy

A total of 282 children in 9 studies were included to analyze the impact of functional electrical stimulation on the walking speed of children with cerebral palsy. See Figure 4 for details. The data showed that the walking speed was increased after functional electrical stimulation compared with the control group (SMD = 0.82, 95%CI = 0.57, 1.07, *Z* = 6.52, *P* < 0.0001). While *I*^2^ = 0%, *P* = 0.5 indicated that there was no significant heterogeneity among the studies. The funnel chart in Figure 5 showed that the literature distribution was uniform and symmetrical, and Begg's test illustrated no publication bias among studies.

### 3.3. Effect of Functional Electrical Stimulation on Walking Steps of Children with Cerebral Palsy

A total of 282 children in 9 studies were included to analyze the impact of functional electrical stimulation on the walking steps of children with cerebral palsy. See Figure 6 for details. The data showed that compared with the control group, the walking step length was increased after functional electrical stimulation treatment (SMD = 1.34, 95%CI = 1.07, 1.60, *Z* = 9.91, *P* < 0.0001). And *I*^2^ = 31%, *P* = 0.17, indicating no significant heterogeneity among the studies. The funnel chart showed that the literature distribution was uniform and symmetrical (Figure 7), and Begg's test indicates no publication bias among studies.

## 4. Discussion

The current research results preliminarily support the use of functional electrical stimulation in treating children with cerebral palsy with walking disorders and activity restriction. The meta-analysis of gait parameters indicated that walking ability was improved after treatment. Our results are consistent with previous studies on functional electrical stimulation to improve gait speed [21]. Therefore, functional electrical stimulation is a feasible treatment for children with cerebral palsy who have difficulty in walking.

The Meta-analysis results showed that the gait speed of children with cerebral palsy has improved after functional electrical stimulation treatment. However, a higher gait speed has dual characteristics. On the one hand, higher gait speed is related to lower gait stability, poor muscle fine control, and joint stiffness. Therefore, children with cerebral palsy may generally adopt compensation strategies to increase gait stability by reducing gait speed and decreasing the risk of falls [22]. Due to the lower instability of walking than the perception threshold of children, children may gradually increase their gait speed when they try to control their gait autonomously, which is also a manifestation of their self-control ability [23]. Here, the gait speed shows a dual explanation. Therefore, it is biased and insufficient to simply explain whether each treatment method effectively improves the gait of children with cerebral palsy from the perspective of gait speed. At this time, it is necessary to refer to the spatial-temporal parameters of gait, including step size analysis, to judge the impact on gait comprehensively. Since walking is a dynamic task, the impairment of motor ability of children with cerebral palsy makes it difficult to maintain balance during dynamic walking. Children need to shorten their steps and reduce the swing of their bodies to sustain gait stability and maintain the center of gravity [24]. When the children's walking ability improves, their ability to maintain the center of gravity is better, and their ability to resist the body swing is stronger. At this time, the children's walking strategy may correspondingly increase the step size and the walking speed. Functional electrical stimulation device application can support muscles or nerves with impaired motor control ability to enhance control and execution during walking [9]. FES is applied in the gait cycle mainly by stimulating the common peroneal nerve and the corresponding calf muscles to correct the gait swing state deviation and improve the walking ability [10]. The meta-analysis results of this study showed that functional electrical stimulation treatment could increase the walking speed of children with cerebral palsy (SMD = 0.82, *P* < 0.0001) and increase the walking step length of children with cerebral palsy (SMD = 1.34, 95%CI = 1.07, 1.60, *Z* = 9.91, *P* < 0.0001). The results indicated that increased walking pace and step lengths could improve the walking ability in children with cerebral palsy.

However, we realize that it is necessary to strengthen the understanding of the etiology and symptoms of cerebral palsy. After all, there are still contradictions among current literature, which requires a sounder basic theory to provide a more convincing explanation for the clinic. Ideally, theoretically unquestionable research can provide the best clinical intervention. This study included the most complete updated evidence-based medical evidence, which might promote the selection of gait treatment measures. After all, functional electrical stimulation devices are small in size and easy to use compared with other devices. Their role in improving gait is also supported by current evidence-based medical evidence. However, the number of high-quality randomized controlled trials of functional electrical stimulation therapy and the number of patients participating in the trials are insufficient. The limited number of literature is also the inadequacy of this paper. Therefore, improving the gait parameters of patients with functional nerve stimulation therapy requires a larger number of patient samples and more in-depth research.

In conclusion, this study compared the effects of the functional nerve stimulation treatment group and control group on improving gait parameters of children with cerebral palsy. The results illustrated an increase in gait speed and step length of children with cerebral palsy after treating with functional nerve stimulation. Therefore, functional nerve stimulation can improve the walking of children with cerebral palsy. Meanwhile, this study needs more research data to determine the benefits. The results of this study may better guide the clinical practice and better use of health and financial resources.

## Figures and Tables

**Figure 1:** Document screening and exclusion process.

**Figure 2:** Summary of study bias risk.

**Figure 3:** Details of bias risk of each study.

**Figure 4:** Forest diagram of walking speed meta-analysis in FES group and control group.

**Figure 5:** Funnel chart of walking speed meta-analysis in FES group and control group.

**Figure 6:** Forest diagram of step size meta-analysis in FES group and control group.

**Figure 7:** Funnel chart of step size meta-analysis in FES group and control group.

## Data Availability

The data used during the current study are available from the corresponding author.
